# Lipid droplets in granulosa cells are correlated with reduced pregnancy rates

**DOI:** 10.1186/s13048-019-0606-1

**Published:** 2020-01-06

**Authors:** Shira Raviv, Shay Hantisteanu, Shilhav Meisel Sharon, Yuval Atzmon, Mediea Michaeli, Einat Shalom-Paz

**Affiliations:** 1 In Vitro Fertilization Department, Hillel Yaffe Medical Center, Hadera, Israel; 2 Obstetrics, Fertility and Gynecology Research Laboratory, Hillel Yaffe Medical Center, Hadera, Israel

**Keywords:** BMI, Cumulus cells, Granulosa cells, Lipid droplets, CRP leve

## Abstract

**Background:**

Lipids are an important source for energy production during oocyte maturation. The accumulation of intracellular lipids binds to proteins to form lipid droplets. This may lead to cellular lipotoxicity. The impact of lipotoxicity on cumulus and granulosa cells has been reported. This pilot study evaluated their correlation to oocyte and embryo quality.

**Design:**

Prospective case-control study.

**Setting**: Referral IVF unit.

**Patients**: Women younger than age 40, undergoing IVF with intracytoplasmic sperm injection.

**Interventions:** 15 women with BMI > 30 (high BMI) and 26 women with BMI < 25 (low BMI) were enrolled. IVF outcomes were compared between groups based on BMI. Lipid content in cumulus and granulosa cells was evaluated using quantitative and descriptive methods. Lipid profile, hormonal profile and C-reactive protein were evaluated in blood and follicular fluid samples. Demographic and treatment data, as well as pregnancy rates were collected from electronic medical records.

**Results:**

Higher levels of LDL and CRP, slower cell division rate and lower embryo quality were found in the group with high BMI. There was no difference in pregnancy rates between groups. In light of these findings, treatment outcomes were reanalyzed according to patients who became pregnant and those who did not. We found that patients who conceived had significantly lower fat content in the granulosa cells, reflected by mean fluorescence intensity recorded by flow cytometry analysis (23,404 vs. 9370, *P* = 0.03).

**Conclusions:**

BMI has no effect on lipid content in cumulus and granulosa cells, and does not affect likelihood of pregnancy. However, women who achieved pregnancy, regardless of their BMI, had lower lipid levels in their granulosa cells. This finding is important and further study is needed to evaluate lipid content in granulosa cells as a potential predictor of IVF treatment success.

## Introduction

Obesity is a worldwide epidemic and a risk-factor for many diseases. The effect of obesity on female fertility has been examined extensively and a significant relation was found between obesity and the reproductive system. Obese women have lower spontaneous pregnancy rates and increased risk for spontaneous abortion. They present with higher incidence of ovulation disorders, and infertility compared to normal weight women. Furthermore, obesity affects the outcome of fertility treatments, resulting in decreased ovarian response to stimulation, lower quantity and quality of oocytes, and adverse effects on the quality of embryos, and on the chances of conception [1–4].

Lipids are an important source for energy production during oocyte maturation, fertilization, and preimplantation development. Cholesterol specifically, plays a significant role as a precursor in the steroidogenic pathway [5] and by that, may adversely affect obese patients. Obesity leads to hyperlipidemia, in which lipids accumulate, and are stored in cells other than adipocytes due to increased cell uptake of fatty acids, triglycerides and cholesterol. The accumulation of intracellular lipids leads to high levels of free fatty acids that cause oxidative damage and produce highly active oxidative metabolites that cause irreversible damage to cells. Prolonged damage and oxidation processes impair the cells’ ability to attain homeostasis and ultimately lead to apoptosis [6]. Excess fatty acids also damage cumulus and granulosa cells, major gonadal functioning cells, and impair their ability to perform normal steroidogenesis [7].

A high fat diet is known to affect the reproductive system and cause ovarian dysfunction regardless of the phenotype. Its effect on ovarian function was irreversible after balancing the diet [8, 9]. The follicular environment influences oocyte growth and quality and thus, its developmental capacity. A study using a mouse model showed that a high-fat diet caused lipotoxicity in granulosa and cumulus cells, which resulted in apoptosis of the cumulus cells. These mice ovulated less often and had lower fertility rates [10]. Another study by Skaznik-Wikiel et al. reported that a high fat diet resulted in a depletion in primordial cells, excess tissue inflammation and accumulation of proinflammatory cytokines, regardless of obesity phenotype [11]. In addition, other studies that evaluated obesity and treatment outcomes, found that high intracellular lipid content in oocytes and embryos impaired cryopreservation [12, 13].

The accumulation of intracellular lipids binds to proteins to form lipid esters, which are the product of the endoplasmic reticulum membrane and are found in the cytoplasm as lipid droplets [14]. Lipid droplet formation is induced by several factors, including long-chain fatty acids, oxidized low-density lipoproteins, oxidative stress, growth factors, inflammatory stimuli, and bacterial infections [15].

Based on the knowledge that a high-fat diet leads to cumulus lipotoxicity in mice and that obesity associated with hyperlipidemia causes damage to human cells, we hypothesized that obesity in women affects granulosa and cumulus cell function, leading to deleterious effects on oocytes and embryos.

This pilot study investigated the correlation between BMI and lipid content in cumulus and granulosa cells and in follicular fluid, and examined the relation between lipid content in granulosa and cumulus cells and fertility outcomes.

## Material and methods

### Study design

Patients were prospectively enrolled from January 2017 to January 2018. This case-control study compared obese patients with BMI > 30 to normal weight controls with BMI < 25 undergoing in vitro fertilization (IVF) with intracytoplasmic sperm injection (ICSI). We recruited patients undergoing ICSI because of the study design and the need for cumulus cells.

### Study participants

Women undergoing IVF with ICSI at the Hillel Yaffe Medical Center were eligible to participate. Additional criteria for study inclusion were age < 40 years, FSH < 12, and more than 4 oocytes collected per patient. Women with BMI > 30 were enrolled into the high BMI group and women with BMI < 25 were enrolled into the low BMI group. Exclusion criteria were age ≥ 40, poor ovarian reserve documented in previous cycles, any adjuvant steroidal treatment to improve ovarian response (DHEA, steroids, etc.) and BMI 25–30.

### Data collection

Patient data collected from electronic medical records included baseline parameters (age, parity, BMI, number of previous IVF/ICSI cycles, and basal FSH), cycle characteristics (length of follicular phase, amount of gonadotropins used, endometrial thickness and estradiol levels on day of hCG administration), clinical outcomes (number of oocytes and mature oocytes, fertilization rate, cleavage rate, blastulation rate, number of transferred embryos and number of frozen embryos) and pregnancy outcomes (chemical pregnancy rate and clinical pregnancy).

### Treatment protocol

Treatment protocols were prescribed according to the physician’s judgment, based on each patient’s characteristics, to prevent compromising the treatment relative to the study goals. The protocols used in this study reflect the normal variety of treatments available in the IVF clinic, as previously described [16]. ICSI was performed for all patients, as previously described [17]. Ovarian stimulation was performed using 150–300 IU of either recombinant FSH (rFSH) (Gonal-Fw, Merck-Serono, Darmstadt, Germany,) or hMG (Menopur, Ferring Pharmaceuticals, Lausanne, Switzerland), with fine-tuning according to age, basal hormone values, antral follicular count at ultrasound and BMI. Estrogen (E2) and progesterone (P) levels were evaluated at every follow-up visit, including the day of hCG (Ovitrelle, Merck-Serono, Darmstadt, Germany,) administration. Ovulation was induced when at least two leading follicles with mean diameter of at least 17 mm were seen. The oocyte was extracted 36 h later.

After oocyte retrieval, IVF or ICSI was performed. Following ICSI, the injected oocytes were placed on EmbryoSlides and incubated in the EmbryoScope™ (Unisense FertiliTech, Aarhus, Denmark) up to 5 days at 37 °C in 5.8% CO_2_ and 5% O_2_. Images of each embryo were acquired every 10 min in seven focal planes, starting from the second polar body extraction up to 120 h after fertilization, to determine the exact timing of cell divisions [18]. Embryos were scored by Known Implantation Data (KID) score and an Alfa ESHRE score, as well as the common morphology [19]. The quality of all available embryos was evaluated and no more than two were transferred on day 3 or one on day 5 of embryonic development. Embryo quality was also evaluated on the day of transfer according to number of cells, symmetry, granularity, type, percentage of fragmentation, presence of multinucleate blastomeres and degree of compaction, as previously described. A top-quality embryo was defined as one with 4–5 cells on day 2 or > 6 equal-size blastomers on day 3, and ≤ 20% fragmentation and no multinucleate cells [20]. The remaining top-quality embryos were vitrified and used in the next frozen embryo transfer, if no pregnancy was achieved in the fresh cycle. The effect of BMI on the number of oocytes retrieved, number of mature oocytes (MII), fertilization and cleavage rates, oocyte diameter, oolema, number of top-quality embryos, and pregnancy rate was compared.

### Collection of follicular fluid and blood samples

On the day of oocyte retrieval, oocytes were separated from the follicular fluid and granulosa cells were filtered and separated from the follicular fluid, as follows. The follicular fluid of all aspirated follicles > 16 mm was collected from both groups of patients on the oocyte retrieval day. Any follicle that was empty or fluid that were mixed with blood were excluded. Blood samples from patients scheduled for oocyte pick-up were obtained.

Before ICSI, upon denudation, cumulus cells were peeled from the oocytes mechanically and with hyaluronic acid. Cumulus and granulosa cells were collected and kept in separate containers for analysis. The follicular fluid was centrifuged at 300 g for 10 min and the supernatant was transferred to a tube and frozen at -80 °C until staining and analysis. The blood samples and the filtered follicular fluid were analyzed for hormone levels including estradiol, progesterone, testosterone, C-reactive protein (CRP), and full lipid profile.

### Measuring hormone levels in plasma and follicular fluid

Progesterone and estradiol levels in the plasma and follicular fluid were measured using electrochemiluminescence ImmunoAssay on ROCHE Cobas 8000, e602. Analytical sensitivity L (0.05 ng/mL), and levels of LH and FSH in the plasma and follicular fluid were measured with Electrochemiluminescence ImmunoAssay on ROCHE Cobas 8000, e602, Analytical sensitivity LOD was 0.1 mIU/mL.

### Pregnancy determination

The β-hCG test was performed 14 days after embryo transfer. Clinical pregnancy and implantation rates were confirmed when a gestational sac with fetal heart beat was visible on ultrasound examination after 7 weeks of gestation. Demographic data, treatment information and results, and pregnancy outcomes were recorded and followed until delivery.

### Isolation of granulosa and cumulus cells

The follicular fluid was filtered through 40 μM strainer to obtain granulosa cells. Clumps of granulosa cells were collected by washing them out of the strainer with cold buffer (PBS + 3% fetal bovine serum). The granulosa cells were centrifuged at 300 g at 4 °C for 6 min. Contaminating red blood cells were lysed by incubating in ACK buffer for 3 min. Cumulus cells were obtained from the IVF lab following oocyte denudation by hyaluronic acid.

### Lipid droplet staining

Granulosa or cumulus cells were re-suspended and fixed in 1% paraformaldehyde at room temperature for 10 min. The fixed cells were washed twice with cold buffer and stained with Nile red (Sigma-Aldrich), a non-specific lipid dyeing material. Nile red solution was prepared by diluting a 1 mg/ml DMSO stock solution by 1:500 in PBS. The fixed cell pellet was re-suspended in 500 μl Nile red solution and incubated at room temperature for 10 min in the dark. Stained cells were washed twice with cold buffer and re-suspended in cold buffer. They were analyzed using flow cytometry (BD LSRII FACS analyzer) to evaluate Nile red levels. The instrument was calibrated with Rainbow beads. The gating strategy was initially set at FSC^hi^SSC^hi^ cells encompassing the large granular granulosa/cumulus cells, followed by gating on FSC-A vs. FSC-H singlet cells. Events collected for granulosa and cumulus samples were 5 × 10^3^–3 × 10^4^ and 5 × 10^3^–2 × 10^4^, respectively.

Mean fluorescence values were determined using Flowjo software. Cells were mounted on glass slides with Prolong Diamond Antifade reagent containing DAPI (Invitrogen) and examined under an epi-fluorescent microscope (Nikon ECLIPSE Ti-S) to evaluate staining specificity and the content of the lipid droplets. Slides were examined at × 20 (object N.A. 0.45) and × 40 (object N.A. 0.6) magnification.

### Statistical analysis

Descriptive statistics in terms of mean, SD, median, percentiles and ranges were performed on all the study parameters. Normal distribution of the quantitative parameters was tested by Kolmogorov-Smirnov test. Based on the results of this test, parametric (t-test) and non-parametric tests (Mann-Whitney U test) were used to evaluate differences between the high BMI and low BMI groups. Differences between groups for categorical parameters were tested with Fisher’s exact test. A receiver operating characteristic (ROC) Youden index statistics curve was used to describe the relationship between the sensitivity and the false positive rate for FACS Nile Red MF-Granulosa cells or for FACS Nile Red MF-Cumulus cells for identifying women who became pregnant vs. those who did not. A multivariate logistic regression model with odds ratios (OR) and 95% confidence intervals (CI) was constructed to predict pregnancy based on several independent parameters including Granulosa cells with the best cutoff (Youden index statistics) form the ROC analysis, BMI in two groups, women’s age, number of oocytes and embryo quality. *P* < 0.05 was considered significant. SPSS, version 25 (SPSS Inc., Chicago, IL) was used for all analyses.

### Ethics approval

The study was conducted at the IVF Unit, Hillel Yaffe Medical Center. The study was approved by the Institutional Review Board and registered (NIH number NCT01672931). All participants provided signed informed consent.

## Results

### Patient characteristics

A total of 41 women were enrolled: 15 with BMI > 30 and 26 with BMI < 25. Age, infertility causes and hormonal profiles were similar between the two groups. The serum LDL level was significantly higher in the high BMI group, as compared to the low BMI group (Table 1).

**Table 1:** Comparable patient’s characteristics

Characteristic	BMI < 25 (*N* = 26)	BMI > 30 (*N* = 15)	*P*-value
Mean BMI (kg/m^2^) mean ± SD; range	22.7 ± 2.4 [17–25]	32.8 ± 2.3 [30–38]	**< 0.0001**
Age, years	32.5 ± 5.4	34.8 ± 4.8	0.18
Primary infertility	13 (50%)	9 (60%)	0.75
LDL cholesterol - blood level (mg/dL)	86.3 ± 28.6	104.9 ± 22.2	**0.048**
Cause of infertility			
Male factor	10 (38.5%)	7 (47%)	0.75
Mechanical factor	4 (15.4%)	2 (13.3%)	1.00
Unexplained	8 (30.8%)	6 (37.5%)	0.73
Anovulation (PCOS)	2 (7.7%)	0	0.52
Hormonal profile			
FSH baseline level (u/L)	7.3 ± 1.6	7.8 ± 1.2	0.25
LH baseline level (u/L)	6.4 ± 2.5	5.6 ± 2.4	0.33
E2 baseline level (pg/dL)	215 [68–826]	161 [43–378]	0.24
E2 level on hCG day (pg/dL)	1744 [1191–2591]	1593 [1302–2164]	0.43

Values are presented as mean ± SD; median 25–75% or ratio (%); Results are considered significant if *P-value* <0.05

Following ovarian stimulation, treatment outcome parameters were compared between the two groups. The number of treatment days, dose of gonadotropins, and final estradiol level on the day of hCG, endometrial thickness, number and quality of oocytes collected, and the fertilization rate were all comparable. We found a significant difference in embryo quality, number of transferred embryos and in the number of available embryos to freeze. However, we did not find any difference in pregnancy rates between the groups (Table 2). Nevertheless, the high BMI group had significantly higher CRP levels in the blood and in the follicular fluid samples, as compared to the low BMI group (Fig. 1).

**Table 2:** Treatment outcomes based on BMI

Variable	BMI < 25 (*N* = 26)	BMI > 30 (*N* = 15)	*P*-value
Total days of treatment	10.2 ± 2.8	11.3 ± 1.7	0.16
Total gonadotropin dose (units)	1350 [1110–1928]	2122 [1240–2434]	0.06
Endometrial thickness (mm)	9.3 ± 1.8	9.7 ± 1.7	0.49
Number of oocytes collected	16.4 ± 10.8	11.3 ± 6.8	0.11
Number of M2 oocytes	9.7 ± 7.1	8.5 ± 6.4	0.61
Number of fertilized oocytes (2PN)	10.4 ± 8.3	7.4 ± 5.1	0.21
Oocyte quality (KID score)	3.8 ± 1.3	3.2 ± 1.6	**0.04**
Number of embryos transferred	1.24 ± 0.93	1.87 ± 0.83	**0.044**
Number of embryos frozen	2 [1–4]	0 [0–2]	**0.03**
Pregnancy / transferred embryos	7/18 (38.9%)	6/14 (42.9%)	1.00
FACS Nile Red MF - Cumulus cells	23,436.44 ± 18,781.44	29,183.00 ± 18,481.69	0.41
FACS Nile Red MF- Granulosa cells	20,995.38 ± 18,455.50	15,354.20 ± 12,261.07	0.46

Values are presented as mean ± SD; median 25–75% or ratio (%); Results are considered significant if *P-value* <0.05

**Fig. 1:** Significantly different CRP levels in the blood and follicular fluid at high and low BMI. Average C-reactive protein (CRP) levels. In the blood (left) and in the follicular fluid (right), according to BMI (low BMI blue, high BMI orange)

### Lipid droplets

Using fluorescent microscopy, we found specific nuclei surrounding droplet-like staining (Fig. 2). Quantification of the Nile Red signal levels in cumulus and granulosa cells by flow cytometry analysis, surprisingly, revealed no difference in the signal between the two BMI groups (Table 2).

**Fig. 2:** Fluorescent microscopy of granulosa and cumulus cells Nile Red staining. Fluorescent microscopy of granulosa and cumulus cells. Lipid droplets (green) are stained with Nile Red and cell nuclei (blue) are stained with DAPI

Next, we reanalyzed the data based on conception outcomes. The cohort was divided into two groups based on conception. Baseline characteristics were comparable (Table 3). Peak estradiol level on pick-up day, in both the follicular fluid and blood samples were higher in patients who eventually underwent successful treatment and achieved pregnancy, HDL was significantly lower and TG were significantly higher in the pregnant group (Table 4). All other clinical parameters were comparable between the pregnant and non-pregnant groups (Table 5). Concomitantly, significantly lower levels of Nile Red staining in the granulosa cells were measured by flow cytometry in patients who eventually conceived (23,404 [15,390-33,401] vs. 9370 [4031-14,675], *P* = 0.03), and a trend was observed in the cumulus cells (38,962 [14119–62,270] vs. 17,270 [12125–20,942]; *P* = 0.09) (Fig. 3, Table 4).

**Table 3:** Comparison of patients’ characteristics based on treatment outcomes

Characteristic	No pregnancy *n* = 25	Pregnancy *n* = 16	*P*-value
BMI	25.6 ± 5.4	27.6 ± 5.6	0.27
AGE	33.2 ± 5.3	33.6 ± 5.3	0.78
Primary infertility	15 (60%)	7 (44%)	0.35
Cause of infertility			
Male factor	12 (48%)	5 (31%)	0.34
Mechanical factor	5 (20%)	1 (6%)	0.38
Unexplained	6 (24%)	8 (50%)	0.10
Anovulation (PCOS)	1 (4%)	1 (6%)	1.00
Baseline hormone profile			
FSH (u/L)	7.2 ± 1.3	7.9 ± 1.7	0.16
LH (u/L)	6.0 ± 2.0	6.1 ± 3.1	0.96
E2 (pg/dL)	176 [68–736]	186 [48–317]	0.55
E2 level on day of hCG treatment(pg/dL)	1642 [1158–2389]	1744 [1325–2694]	0.27

Values are presented as mean ± SD, median 25–75% or ratio (%): Results are considered significant if *P-value* <0.05

**Table 4:** Follicular and blood parameters by pregnancy outcome

Parameter	No pregnancy *n* = 25	Pregnancy *n* = 16	*P*-value
E2-follicular fluid on OPU day (pg/dL)	183,225 [123427–263,082	418,271 [325117–520,939]	**0.012**
E2-Blood on OPU day (pg/dL)	822.6 [577.6–1280]	1208.0 [836.6–1826.5]	**0.05**
CRP-follicular fluid (mg/dL)	0.9 [0.15–3.4]	2.4 [0.52–6.05]	0.25
CRP-Blood (mg/dL)	4.2 [1.1–8.7]	4.9 [2.7–8.1]	0.49
TG-Blood (mg/dL)	98.7 ± 37.5	143.2 ± 57.6	**0.018**
HDL-Blood (mg/dl)	51.3 ± 12.7	42.5 ± 7.8	**0.018**
FACS Nile Red MF Cumulus cells	38,962 [14119–62,270]	17,270 [12125–20,942]	**0.09**
FACS Nile Red MF Granulosa cells	23,404 [15390–33,401]	9370 [4031–14,675]	**0.03**

Values are presented as mean ± SD, range, median 25–75%: Results are considered significant if *P-value* <0.05

**Table 5:** Treatment parameters based on outcomes

Parameter	No pregnancy *n* = 25	Pregnancy *n* = 16	*P*-value
Total days of treatment	10.1 ± 2.1	11.4 ± 2.9	0.12
Total gonadotropin dose (units)	1700 [1143–2162]	1500 [1100–2434]	0.95
Endometrial thickness (mm)	9.5 ± 2.15	9.4 ± 0.96	0.96
Number of oocytes collected	13.7 ± 8.9	15.9 ± 11.1	0.49
Number of M2 oocytes	8.2 ± 4.2	11.0 ± 9.5	0.21
Number of fertilized oocytes (2PN)	8.2 ± 7.1	11.0 ± 7.6	0.25
Oocyte quality (KID score)	3.46 ± 1.5	3.68 ± 1.4	0.32
Number of embryos transferred	1.46 ± 0.98	1.50 ± 0.89	0.89
Number of embryos frozen	1 [0–3.8]	2 [1–3.5]	0.29

Values are presented as mean ± SD, median 25–75% or ratio (%): Results are considered significant if *P-value* <0.05

**Fig. 3:** Nile Red staining of cumulus and granulosa cells. **a** Cumulus cells forward to side scatter plot analysis of pregnant and non-pregnant patients. **b** Histogram analysis of Nile red staining showing fewer lipid droplets in the cumulus cells of a pregnant patient. **c** Granulosa cells forward to side scatter plot analysis of pregnant and non-pregnant patients. **d** Histogram analysis of Nile red staining showing fewer lipid droplets in the granulosa cells of a pregnant patient

### Clinical outcomes

The morphokinetics of the embryos according to BMI are shown in Fig. 4. Patients with higher BMI had longer duration of cell cleavage from the stage of polar body appearance to cell division 4, 4 cells embryos. This morphokinetics timing also influenced the embryo scores, as presented in Table 2. Embryo quality and quantity were significantly lower in the high BMI group, as compared to the low BMI group (Table 2).

**Fig. 4:** Morphokinetics parameters of embryos in the BMI < 25 and BMI > 30 groups. The morphokinetics of embryos according to BMI, Y-axis: duration of cell division. X axis: cleavage point. (BMI < 25 blue, BMI > 30 orange). Patients with BMI > 30 had longer duration of cell cleavage from the stage of polar body (PB) appearance until cell division 4

ROC analysis was used to predict the cutoff of lipid content in the granulosa and cumulus cells. We found that lipid droplet levels < 18,228.5 were correlated with positive pregnancy test. BMI and the accumulation of lipids in granulosa cells with the above cutoff were used in a multivariate model to predict clinical pregnancy. This model revealed that only BMI and lipid accumulation in granulosa cells predicted pregnancy rate. Higher BMI reduced the chance for pregnancy with (OR = 0.035; *P* < 0.0001 and 95% CI (0.007 to 0.16)). Lower stain uptake of granulosa cells increased the chance for pregnancy (OR = 26.2; *P* < 0.0001 and 95% CI (5.3 to 128.9)). All other parameters included in the model, such as age, number of oocytes and embryo quality had no significant effect on conception or pregnancy outcomes.

## Discussion

This study evaluated the impact of BMI level on lipid accumulation in the female gonads, represented by both granulosa and cumulus cells. Although our data revealed no direct correlation between BMI and lipid droplet accumulation and clinical outcomes, we found an increase in fluorescence, possibly resulting from an increase in the number and size of lipid droplets, which was significantly associated with lower pregnancy rates. This also correlated with lower estradiol levels in the follicular fluid and in the blood on OPU day.

Based on our previous study, which reported that smaller oocytes were obtained during IVF treatment in obese patients [21], we examined the correlation between BMI and lipid accumulation in cumulus and granulosa cells. To the best of our knowledge, this is the first study that links obesity, lipid droplets and embryo development in the lab.

We assumed that the follicular fluid, which is an important component in oocyte development (serving as the microenvironment of the growing oocyte) and is an ultra-filtrate of the blood, would reflect the differences between high BMI and low BMI. In fact, we found no direct correlation between BMI to pregnancy outcome; however, a significant difference was seen between high and low accumulation of lipid droplets in cumulus and granulosa cells. This finding may reflect the impact of high fat dietary consumption.

CRP is an acute phase marker, produced by the liver in response to pro-inflammatory cytokines. A strong correlation was shown between serum and follicular fluid CRP levels and higher BMI [22]. This correlation might be associated with chronic anovulation and lack of conception in women undergoing fertility treatments [23, 24]. High CRP levels are characteristic of increased inflammation and oxidative stress [25], which have a strong influence on oocyte development and subsequent embryo quality [26]. The current study found significantly higher CRP levels in the blood and follicular fluid in the high BMI group, as compared to the low BMI group. Thus, our results agree with those of the above studies and with Rebecca et al. [27] who revealed that differences in the ovarian follicular environment might be associated with poorer reproductive outcomes in patients with high BMI. Valckx et al. also showed that metabolic changes in the groups are reflected in the follicular fluid and may affect oocyte quality. However, as in our study, overall, the direct impact of BMI were weak [28].

Embryologists use embryo morphokinetics to establish development models to improve accurate selection of viable embryos. These morphokinetic models are based on several parameters, including the duration between fertilization and each cleavage stage, and were found to be important in the decision of which embryo to use for transfer. In our study, the morphokinetics of the embryos from the high BMI group had significantly slower cleavage. This group also had poorer embryo quality [29]. Our findings are in agreement with previous data that demonstrated faster cleavage achieves more clinical pregnancies and that embryos that develop more quickly seem to exhibit more developmental potential [30].

In agreement with other studies, our data show that the group of patients with high BMI demonstrated a trend toward consistently worse outcomes in terms of peak estradiol level, number of oocytes collected, total M2 oocytes, and fertilization rate. Importantly, more embryos were transferred per cycle and fewer were available for cryopreservation in the high BMI group [31–33]. However, in this study, there was no significant difference in the likelihood of a successful pregnancy between patients with high BMI or low BMI. Several studies targeted the issue that high fat diet, even without obesity, is likely to induce metabolic and reproductive dysfunction. Therefore, this might explain our lack of significant results when comparing pregnancy outcomes between the two BMI groups. It is important to consider that high fat diet alone can result in impaired fertility, even among lean individuals [8].

As steroidogenic cells, the granulosa and cumulus cells need a constant supply of cholesterol as a precursor for conversion to steroids [34]. In the ovaries and adrenal glands, the preferred pathway for steroid production is from lipid droplets which transfer to mitochondria [35]. When we compared the group of patients who conceived and those who did not, both were comparable in terms of patient characteristics. However, we found significantly higher E2 levels in the plasma and follicular fluids of patients who conceived, and significantly lower lipid droplets levels in granulosa and cumulus cells. This might be due to higher consumption of lipids and cholesterol in the high E2 group that achieved pregnancy.

Studies using animal models of obese mice demonstrated marked differences from normal weight mice. The obese mice lacked corpora lutea, follicular atresia rate was higher, they had excessive accumulation of lipid droplets in follicular cells and in oocytes and had mitochondrial damage [36, 37]. The conclusion was that excessive lipid storage causes disorders of ovarian function in obese mice and that local lipid overload leads to advanced follicular atresia, with apoptosis and defective steroidogenesis by decreased StAR protein production.

Another mechanism suggested to influence lipid metabolism is hormone-sensitive lipase (HSL). HSL is a key enzyme for the mobilization of fatty acids from acylglycerols in adipocytes, as well as non-adipocytes [38] . HSL knockout mice exhibit azoospermia. Wang et al. demonstrated higher cholesterol content in HSL knockout mice testis [39]. It is possible that a reduction in HSL protein and/or activity was the mechanism in our group of patients who did not achieve pregnancy and who had higher lipid quantity in granulosa and cumulus cells.

Our data revealed significantly lower peak estradiol levels in patients with high BMI vs. low BMI; however, we could not demonstrate differences in lipid droplet accumulation. This might become apparent with larger sample sizes. Higher fluorescence, which might be due to larger number or size of lipid droplets, was found in granulosa and cumulus cells among the patients who did not conceive. They also had lower peak estradiol levels, which might imply ovarian dysfunction and abnormal steroidogenesis in this group. As was reported and discussed in previous studies and in animal models, the obese phenotype might have less of an effect on ovarian function than diet does [8].

This was a prospective study that integrated basic science laboratory research with clinical outcomes. However, we want to point out some weaknesses, as well. The number of participants was relatively small, as this was a pilot study. Further insights may be obtained by increasing the sample size; for example, re-assessing the cutoff of the lipid droplet levels and correlations with pregnancy rates, the correlation between lipid droplets and BMI as a continuous parameter and the impact of diet on lipid content in the cells, and the impact on pregnancy outcomes.

## Conclusions

Based on the above findings, demonstrating poorer IVF-ICSI treatment outcomes and lower pregnancy rates among patients with higher lipid droplets in their cumulus and granulosa cells, we recommend lifestyle changes for patients who are above the normal weight range. Although we were not able to demonstrate a significant effect of BMI per se on pregnancy rates, this study found a significant association between high accumulation of lipid droplets and clinical outcomes in IVF treatment. Our results could not explain the overall effect of BMI on IVF treatment outcomes. However, the effect of accumulation of lipid droplets in granulosa and cumulus cells, potentially derived from diet had an impact on treatment outcomes. Therefore, we want to emphasize the importance of diet beyond BMI. It is well-established that obesity predisposes women to several general and obstetrical complications during pregnancy and delivery [40–42]. Therefore, it is important to discuss fertility and pregnancy complications prior to conception, with patients who have high BMI [43, 44]. Further studies are needed to elucidate the exact molecular mechanisms associated with these findings.
